# Documentation of Herbal Medicines Used for the Treatment and Management of Human Diseases by Some Communities in Southern Ghana

**DOI:** 10.1155/2017/3043061

**Published:** 2017-06-08

**Authors:** Augustine A. Boadu, Alex Asase

**Affiliations:** Department of Plant and Environmental Biology, University of Ghana, P.O. Box LG 55, Legon, Ghana

## Abstract

Traditional medicine is an important component of the health care system of most developing countries. However, indigenous knowledge about herbal medicines of many Ghanaian cultures has not yet been investigated. The aim of the present study was to document herbal medicines used by traditional healers to treat and manage human diseases and ailments by some communities living in Ghana. The study was conducted in eight communities in southern Ghana. Data were collected from 45 healers using ethnobotanical questionnaire and voucher specimens were collected. A total of 52 species of plants belonging to 28 plant families were reportedly used for treatment and management of 42 diseases and ailments. Medicinal plants were commonly harvested from the wild and degraded lowland areas in the morning from loamy soil. Herbal medicines were prepared in the form of decoctions (67%) and infusions (33%). Oral administration of the herbals was most (77%) common route of administration whereas the least used routes were nasal (1%) and rectal (2%). The results of the study show that herbal medicines are used for treatment and management of both common and specialized human diseases and that factors of place and time are considered important during harvesting of plants for treatments.

## 1. Introduction

According to the World Health Organization (WHO) about 80% of developing countries depend on traditional medicines for their primary health care needs [1]. In Ghana, traditional medicine, particularly herbal medicines, is an important component of the health care system of the people [2]. The utilization of herbal medicines and associated medicinal plants in Ghana has been documented by many authors [e.g., [3–5]] although there are still many indigenous cultures and communities in Ghana that possess a great store of traditional knowledge about herbal medicines for treatment of various human ailments, which are yet to be documented. The use of herbal medicine in Ghana is widespread but highly diverse due to floristic and cultural diversity, and traditional medicine has huge impacts on the local economy and biodiversity conservation. The rich history of use of herbal medicines and innovative utilization of plants as sources of medicines in Ghana, and broadly within Africa, has been passed down through generations largely as oral tradition [6] and as such it is important that this knowledge be documented. The WHO has a keen interest in documenting the use of medicinal plants by indigenous people from different parts of the world [7].

Documentation of indigenous knowledge about utilization of medicinal plants is important for a plethora of reasons. Firstly, it ensures that indigenous culture heritage is preserved from being lost for the use of both present and future generations [8]. Studies have indicated that indigenous knowledge about herbal medicines is continuously being lost through factors such as acculturation and biodiversity losses. For example, a comparative study of contemporary plant uses in Ghana shows that the* materia medica* of the Fanti, Ga, and Ashanti has changed considerably over time [6]. Secondly, through further research such as phytochemical, biochemical, pharmacological, and clinical studies information on indigenous herbal medicines can lead to discovery of new bioactive agents for treatment of ailments. Despite the recent interest in molecular modelling, combinatorial chemistry, and other synthetic chemistry techniques by pharmaceutical companies and funding organizations, natural products, and particularly medicinal plants, remain an important source of new drugs, new drug leads, and new chemical entities (NCEs) [9, 10]. Thirdly, biodiversity conservation can be enhanced when information about plants that are harvested and utilized in the management of ailments within particular areas are available [3]. For biodiversity conservation, it is also important to know what quantities of plant materials are harvested, not only for home consumption but also for trade. Commercial trade often stimulates extensive wild-collection, which often has negative effects on medicinal plant population sizes and recovery after harvesting. On the other hand, the trade and marketing of herbal medicine creates employment for thousands of people, for example, in Ghana [11]. For these reasons, the harvest should be documented and sustainable so this can continue to be a profitable resource for future generations [12].

The aim of this study was to investigate herbal medicines commonly used for the treatment and management of human diseases and ailments by some communities living in southern Ghana. To the best of our knowledge no specific previous ethnobotanical report on use of herbal medicines as yet exists for the studied communities. Here, we investigated aspects of the diversity and harvesting of medicinal plants as well as the modes of preparation and routes of administration of the herbal medicines. It is hoped that this baseline data will, in addition to preservation of indigenous knowledge, generate interest for studies regarding the harvesting patterns, bioactivity, and safety of the medicinal plants being used. Specifically, our study addressed the following questions: (1) What are the most important species and families of plants being used? (2) Which plant parts are most frequently used? (3) Which diseases are commonly treated with the herbal medicines? (4) What is the percentage of plants that are used for treatment and management of a single disease versus multiple diseases? (5) Which factors of place and time are considered important during harvesting of plants for treatments? (6) What are the most common methods of preparation and routes of administration of the herbal medicines? We hypothesize that healers are consulted for herbal medicines for the treatment and management of only specialized human diseases/ailments. We further hypothesize that factors of place and time are considered important during harvesting of individual plants for treatments and management of human diseases by traditional healers.

## 2. Materials and Methods

### 2.1. Study Area

The present study was conducted in 8 communities located within Akuapim-North Municipality and Lower Manya-Krobo Municipality in southern Ghana (Figure 1). Selection of the studied communities was based on preliminary surveys by the first author, which showed that traditional healers in the communities possess rich but undocumented traditional knowledge about use of herbal medicines. The selection of the communities was also based on the perceived willingness of healers in the communities to cooperate with the objectives of our study.

The Akuapim-North Municipality covers a land area of ca. 450 km^2^ and is located on longitude 6°1′N and latitude 0°50′W and at altitude 408 m above sea level. The major vegetation type is semidecidous forest and the area is mountainous consisting of the Togo-Atakora hills. There are two raining seasons—a major rainfall between May and August and the minor rainfall in October. Average annual rainfall is about 1250–1270 mm and mean daily temperatures range between 25 and 30°C (http://www.statsghana.gov.gh). The natives are the Akuapim people although other ethnic groups are common in the area. Christianity is the predominant religion in the area.

Lower Manya-Krobo Municipality is located between latitudes 6°05′N and 6°30′N and longitudes 0°8′W and 0°20′W, with an altitude of 457.5 m above sea level. The vegetation is semidecidous forest with patches of savanna woodland and dispersed secondary forests. The municipality lies within the semiequatorial climate belt with mean annual rainfall between 9000 and 11500 mm. Temperatures are usually high ranging between 26 and 35°C. Topography is relatively flat with isolated hills (http://www.statsghana.gov.gh). The native people of the area are Krobo but there are people from other ethnic groups such as Ewes, Akans, and Hausas. The majority of people are Christians with few Muslims and Traditionalists (http://www.statsghana.gov.gh).

### 2.2. Selection of Healers and Data Collection

The present study was conducted following the guidelines of the Code of Ethics of the International Society of Ethnobiology [13]. A total of 80 healers from the study area were initially approached through peer recommendations. The purpose of the study including research objectives, methods of data collection, and intention to publish data were thoroughly explained to each individual healer that was approached. Subsequently, detailed interviews for purposes of data collection were carried out with only healers that agreed to participate in the study and have signed an individual written prior informed consent. Data were collected from 45 traditional healers (Table 1) through interviews using semistructured questionnaire with predetermined open-ended and direct questions [14]. The interviews were based on the plants being used, diseases and ailments treated, modes of preparation and administration of the herbal remedies, and factors of time and place that they consider as important when harvesting medicinal plants. Healers were interviewed individually, and the interviews were mostly conducted in their homes and places where they collected plants for treatments.

### 2.3. Specimen Collection and Plant Identification

Plant specimens were collected with the healers interviewed in places where they normally collected plant materials for use, pressed, and processed following standard ethnobotanical practices [15]. Plant identification was achieved by matching local names with those in standard literature [16] following the work of [17] as well as by comparison of the voucher specimens collected with those in the Ghana Herbarium at Department of Plant and Environmental Biology, University of Ghana. Classification and names of plants were authenticated using The Plant List (2013) database (http://www.theplantlist.org).

## 3. Results and Discussion

### 3.1. Composition of Herbal Medicines

In total, 52 species of plants belonging to 28 plant families were documented (Table 2). Of the 28 families of plants, members of the Fabaceae, Euphorbiaceae, Asteraceae, and Sapindaceae were the most commonly used ones (12% in each case) in the herbal medicines (Figure 2(a)). The use of members of the above families in herbal medicines is widely known in Ghana [3]. It is widely known that members of the families contain secondary metabolites such as tannins, phenolics, and alkaloids that are responsible for their bioactivity.

Trees formed the majority (37%) of the plants being used (Figure 2(b)). Two of the species of plants reported being used, namely,* Pteridium aquilinum* (L.) Kuhn and* Pteridium esculentum* (Forst.) Nakai, were ferns whereas the rest of the plants were vascular plants. There is very little information on the use of ferns in the Ghanaian traditional pharmacopeia [see, e.g., [3, 4]]. Species most commonly reported being used were* Aloe vera* L. and* Paullinia pinnata* L. with a percentage frequency of citation 7% each out of a total of 92 citations. About 54% of the species reported being used were cited only once by the healers during the period of the current study.

Leaves formed 57% of the herbal medicines documented. Other plant parts used were fruits, barks, and whole plants (Figure 2(c)). Leaves are commonly used in herbal medicines because they represent the site of most photosynthetic activity in plants and they also contain very high concentrations of secondary metabolites. The benefit of a high proportion of leaves being used is also that the threat posed to the populations of the plant community is minimal compared to harvesting of roots and barks. The use of a combination of various plants parts formed 18% of the herbal medicines and this use is well documented in the literature. Since the composition of secondary metabolites differs in plant organs [18], the use of different organs of the same plant in the herbal medicines might be to ensure extraction of the different bioactive agents.

### 3.2. Common Human Diseases and Ailments

Herbal medicines were reportedly used for treatment and management of 42 diseases and ailments. Two or more herbal medicines were reportedly used for treatment and management of 17 the diseases and/ailments, and the herbals were most commonly used for treatment and management of stroke, fevers, and diabetes (Figure 3). The herbal medicines were used for treatment and management of both common ailments (e.g., cuts, foot root) as well as the more specialized diseases such as stroke, diabetes, cancer, and stomach ulcer. Some of the diseases such as stroke, malaria, and HIV/AIDS are among the top 10 causes of deaths in Ghana (https://www.cdc.gov/globalhealth/countries/ghana/). Knowledge of frequently reported diseases and/ailments can be an indication of health care issues in a region and it should be of great importance to health care organizations and government.

About 43% of the species of plants were reportedly used in treatment of a single disease whereas the rest of the plants (57%) were involved in treatment of more than one disease/ailment. Medicinal plants are commonly used in the management of different ailments because they contain a variety of bioactive agents such as alkaloids and terpenoids [18, 19]. It is possible to isolate the bioactive agents or compounds from extracts made from plants for detailed pharmacological and clinical investigations to be made. Nevertheless, in some cases isolation of bioactive agents has been unsuccessful even though the extracts are active. In the latter case, characterization of the active extract could enable structure-related activity studies leading to possible synthesis of a more potent drug to be developed.

### 3.3. Harvesting of Plant Materials

Almost all the healers (98%) interviewed harvested plant materials from lowland areas (Table 3). About half of the healers harvested plant materials from forest-mosaic vegetation type while 7% of the healers considered vegetation type unimportant when harvesting plants. About 93% of the healers considered the habitat of individual plants as important during harvesting. Of the healers who considered habitat as important, 44% harvested plants from the wild, and 36% harvested from degraded areas and few (13%) of them harvested plants from their home gardens. The values of degraded/secondary habitats [20] and home gardens [21, 22] as sources of medicinal plants have been discussed by authors. Secondary forests are gaining more importance for medicinal plant collection as old-growth forests are becoming scarce and overexploited [23, 24]. Our result is similar to that of [25], which indicated that healers favoured primary forest and wild habitats in terms of medicinal plant collection. According to [26] if a plant grows readily in the wild and produces a good yield of active constituents or takes several years to mature then collection from the wild is most practicable. On the other hand, if plants that are harvested from wild vegetation are rare or have endemic status, overharvesting can be a particularly serious threat [27]. About 76% of the healers harvested plants from loamy soils and 18% from sandy soil. None of the healers harvested plants from clayey soils while about 6% of the healer did not consider soil type when harvesting plants. Healers did not explain why they avoided clayey soil and we did not find any scientific evidence that clayey soil plants do not produce pharmacologically active secondary metabolites. Soil physiochemical properties, particularly nutrient levels, affect growth and development of plants. The levels of secondary metabolites in plant tissues vary with resource availability [28], and plant nutrient balance in soil is thought to influence production of secondary compounds at the level of metabolic regulation in plants [29]. Topography of an area affects rainfall, soil type, and amount of light reaching a plant and therefore indirectly also affects plant growth and development. In this study, about 91% of the healers harvest medicinal plants in areas of flat topography while about 9% of the healers harvested plants from areas of gentle slope.

The time of harvesting medicinal plants was investigated with respect to time of day (24 hr. duration) and season (dry versus wet season) of the year. About 57% of healers harvested plants in the morning followed by 28.9% who collected plants anytime of the day and then 4.4% that collected plants in the afternoon. None of the healers collected plant materials in the night and about 9% considered time of the day unimportant when harvesting plant materials for herbal preparations. Plants materials were harvested in the morning because of the importance of healthcare to healers as they collected plants first thing in the day. About 28% of the healers harvested plants anytime of the day, which might suggest that healers also collected plants as when they are needed. According to the healers they collected plants any time of the day because they sometimes needed to treat emergency cases. There is scientific evidence to support the fact that yield of some plant chemical constituents differs within a time span of 24 hours due to the interconversions of compounds [19]. According to [30], time of the day should be given important consideration when collecting medicinal plants in order to obtain optimum yield of desired products. For season of the year, more than half of the healers (67%) harvested plants during both dry and wet seasons followed by 20.0% who collected in only the wet season and about 7% collected in only dry season. About 7% of the healers did not consider season of the year as an important factor during harvesting of plant materials although the availability of certain plant parts could be directly related to season of the year.

### 3.4. Methods of Preparation and Administration of Herbal Medicines

The harvested plant materials were used in preparation of 81 herbal medicines mainly in the form of decoctions (67%) and infusions (33%). Although it is documented that a variety of methods have been used for preparation of herbal medicines the methods of decoctions and infusions have been the widely reported [e.g., [18]]. However, differences exist in the preparations of decoctions and infusions both within healers and from place to place. In the study area, diversity existed among healers in the amount of menstruum (mainly water), length of time of boiling, and how long the decoctions were kept. Infusions were made by adding water/local gin (akpeteshie) to the pulverized plant materials although the amount of solvent added and duration of use of infusions differed. Generally, there were no standards in the methods of preparation of the herbal medicines by even the same healer and this lack of standardization is a major disadvantage of traditional medicine [26, 31]. It also means that herbal medicines made by the same healer could vary in potency, which has implications in their use for treatment of patients.

The routes of administration of the remedies reported in this study were oral, rectal, topical, and nasal (Table 1). However, the most common route of administration was oral (77%) followed by a combination of oral and topical routes (10%) whereas the least used routes were nasal (1%) and rectal (2%). The fact that oral route of administration of the herbals was most common was not a surprise as this has been previously reported [18, 32]. However, a recent study in [33] found frequent use of herbal enemas (rectal) in Western African traditional medicine. The route of administration of herbal medicines could be related to bioactive agents in the extracts of the plants [32]. For example, herbal medicines whose bioactive agents are alkaloids are easily assimilated when administered orally while terpenoids especially essential oils are best administered through dermal and/nasal routes. Both decoctions and infusions were mostly administered orally, 45% and 17%, respectively. Only infusions were administered via the rectal and nasal routes.

## 4. Conclusions

In this paper, we have documented the current state of knowledge and use of herbal medicines for treatment and management of human diseases among some communities living in southern Ghana. This documentation contributes primary data to the wealth of data stored on the indigenous knowledge on medicinal plants from Ghana. The findings from the study suggest that healers are consulted for herbal medicines for the treatment and management of both common and specialized diseases and ailments. The extent to which the people living in the area consult the healers is unknown but it is important to understanding this in order to determine the proper role of herbal medicine in the health care system of the people. It is also essential to scientifically evaluate the specific uses of the medicinal plants reported in the current study using plant materials from the area through pharmacological, toxicological, and clinical studies in order to ensure the safety of the people consuming the medicines and for possible drug development. The results of the study have also confirmed that factors of time and place are given considerations during harvesting of plant materials by healers. Further studies on the methods and quantities of plant materials that are harvested for treatment will improve our understanding on the impacts of harvesting of medicinal plants on biodiversity conservation in the area.

## Figures and Tables

**Figure 1:** Map of study area showing communities where study was conducted.

**Figure 2:** Composition of herbal remedies used in terms of (a) plant families, (b) habit of plants, and (c) percentage of plant parts.

**Figure 3:** Human diseases commonly treated and/managed with herbal medicines.

**Table 1:** Biodata on traditional healers interviewed.

Categories	Variables	Number of healers	Percentage of healers
Sex	Female	13	28.9
	Male	32	71.1

Religion	Christians	37	82.2
	Traditionalist	8	17.8

Formal education	None	6	13.3
	Basic	30	66.7
	Secondary	9	20.0

Age-groups	40–49	11	24.4
	50–59	10	22.2
	60–69	10	22.2
	70–79	9	20.0
	80–89	4	8.9
	≥90	1	2.2

Years of practice	10–19	2	4.4
	20–29	11	24.4
	30–39	11	24.4
	40–49	15	33.3
	50–59	5	11.1
	≥60	1	2.2

**Table 2:** Species of plants reportedly being used by healers arranged according to their families with information on their habits, ailments treated, plant parts used, methods of preparation, and route of administration of the plants.

Families	Scientific names (voucher specimen #)	Local names (Akuapem/Krobo)	Frequency of citation (%)	Habit of plant	Diseases and/ailments	Plant parts	Methods of preparation	Route of administration
Acanthaceae	*Ruellia brevifolia* (Pohl) C. Ezcurra (A029)	Mokotso (Krobo)	1.1	Herb	Halitosis	Leaf	Infusion	Nasal

Aloaceae	*Aloe vera* L. (A001)	Aloe	6.5	Herb	Diabetes Diabetes Typhoid fever Baldness	Leaf Leaf Leaf Leaf	Decoction Decoction Infusion Decoction	Oral Oral Oral Topical

Amaranthaceae	*Alternanthera pungens* Kunth. (A028)	Nkassenkasee (Akuapem)	1.1	Herb	Stomach ulcer	Whole plant	Infusion	Rectal

Annonaceae	*Polyalthia longifolia* (Sonn.) Thwaites (K001)	Tsogaga (Krobo)	2.2	Tree	Fever	Leaf	Decoction	Oral

Apocynaceae	*Alstonia boonei* De Wild. (A026)	Nyamedua (Akuapem)	1.1	Tree	Sexual disorders	Root and bark	Infusion	Topical
	*Rauvolfia vomitoria* Wennberg (A025)	Unknown	1.1	Tree	Osteoarthritis	Leaf and bark	Infusion	Rectal

Asclepiadaceae	*Calotropis gigantea* (L.) W. T. Aiton	Unknown	1.1	Shrub	Heart burns	Leaf	Decoction	Oral

Asteraceae	*Chromolaena odorata* (L.) R. M. King (K003)	Acheampong (Akuapem/Krobo)	3.2	Shrub	Typhoid fever Stop bleeding Typhoid fever	Leaf Leaf Leaf	Decoction Decoction Infusion	Oral Oral Oral
	*Launaea taraxacifolia*. (Wild). Amin ex. C. Jeffrey (K002)	Unknown	3.2	Herb	Blood pressure Diuretic Blood pressure	Leaf Leaf Leaf	Infusion Decoction Infusion	Oral Oral Oral
	*Vernonia amygdalina* Delile (A023)	Awunyun (Akuapem)	3.2	Shrub	Malaria	Whole plant	Infusion	Oral
	*Vernonia conferta* Benth. (K010)	Owudifukete (Akuapem)	2.2	Shrub	Diabetes	Root and bark	Decoction	Oral

Bignoniaceae	*Kigelia africana* (Lam.) Benth. (K004)	Nfuten (Akuapem)	1.1	Tree	Piles	Bark	Infusion	Oral
	*Spathodea campanulata* P. Beauv. (K005)	Akuakua nisuo (Akuapem)	1.1	Tree	Stroke	Leaf	Decoction	Oral

Bombacaceae	*Bombax buonopozense* P. Beauv. (A002)	Nyankuduro/Akonkodies (Akuapem)		Tree	Stroke Diabetes	Leaf Leaf	Decoction Infusion	Oral Oral/Topical

Boraginaceae	*Heliotropium indicum* L. (K007)	Akomfemtikoro (Akuapem)	2.2	Herb	Convulsion	Leaf	Infusion	Oral

Capparidaceae	*Euadenia eminens* L. (K008)	Dinsikuro (Akuapem)	1.1	Herb	Low sperm count	Root and bark	Decoction	Oral

Chrysobalanaceae	*Maranthes robusta* (Oliv.) Prance (K009)	Afambere (Akuapem)	1.1	Tree	Rheumatism	Leaf and seed	Decoction	Oral/Topical

Combretaceae	*Terminalia superba* Engl. & Diels (A021)	Ofram (Akuapem)	1.1	Tree	Convulsion	Root and bark	Decoction	Oral/Topical

Cucurbitaceae	*Momordica charantia* L. (K020)	Nyenye (Krobo)	2.2	Climber	Snake bite Diabetes	Whole plant Whole plant	Infusion Decoction	Oral Oral

Cyperaceae	*Cyperus esculentus* L. (A020)	Winto/Wintino (Krobo)	1.1	Herb	Typhoid fever	Whole plant	Decoction	Oral

Dennstaedtiaceae	*Pteridium aquilinum* (L.) Kuhn (A012)	Unknown	1.1	Herb	Fever	Leaf	Decoction	Oral
	*Pteridium esculentum* (Forst.) Nakai (A018)	Meyaabea (Akuapem)	1.1	Herb	Menstrual disorders	Leaf	Decoction	Oral

Euphorbiaceae	*Bridelia ferruginea* Benth (K014)	Unknown	1.1	Tree	Diarrhoea	Root	Decoction	Oral
	*Discoglypremna caloneura* (Pax) Prain (A017)	Unknown	2.2.	Tree	Stroke Female infertility	Leaf and root Leaf and root	Decoction Decoction	Oral Oral/Rectal
	*Drypetes aubrevillei* Leandri (K017)	Duameko (Akuapem)	1.1	Shrub	Stroke	Root	Decoction	Oral/Topical
	*Drypetes floribunda* Hutch. (K016)	Katirika (Akuapem)	1.1	Shrub	Miscarriage	Root and bark	Decoction	Oral
	*Jatropha curcas* L. (A014)	Unknown	1.1	Shrub	Hernia	Leaf	Infusion	Oral
	*Jatropha gossypifolia* L. (A015)	Unknown	1.1	Shrub	High fever	Leaf and fruit	Decoction	Oral
	*Macaranga barteri* Müll. Arg. (K015)	Opam (Akuapem)	1.1	Shrub	Foot rot	Bark	Decoction	Oral
	*Uapaca guineensis *Müll. Arg. (A016)	Agyahere (Akuapem)	1.1	Tree	Stroke	Root, bark and leaf	Decoction	Topical

Fabaceae	*Acacia senegalensis* (Houtt.) Roberty (K022)	Unknown	1.1	Tree	High fever	Leaf	Decoction	Oral
	*Albizia ferruginea* (Guill. & Perr.) B. (K021)	Awiemtosamina (Akuapem)	1.1	Tree	Diarrhoea	Root	Decoction	Oral
	*Baphia nitida* Lodd. (A005)	Odwaen	1.1	Shrub	Retarded growth	Leaf	Infusion	Topical
	*Berlinia* sp. (A013)	Unknown	2.2	Tree	Rheumatism Fever	Root and bark Bark	Infusion Decoction	Topical Oral
	Cassia alata L. (K023)	Kobatso (Krobo)	3.3	Shrub	Purgative Menstrual disorders Fertility problems	Leaf Leaf Leaf	Decoction Decoction Decoction	Oral Oral Oral
	*Copaifera salikounda* Heckel (A030)	Otedua (Akuapem)	2.2	Tree	High fever Piles	Bark Root and bark	Decoction Decoction	Topical Oral/Rectal

Lamiaceae	*Ocimum gratissimum* Seem. (A011)	Nunnum (Akuapem)	2.2	Herb	Bloating	Leaf	Infusion	Oral/Topical

Malvaceae	*Gossypium hirsutum* L. (K024)	Asawadua (Akuapem)	2.2	Herb	Osteoarthritis Infertility	Leaf Leaf	Infusion Infusion	Oral Oral

Meliaceae	*Azadirachta indica* A. Juss (A008)	Nimtso (Krobo)	5.4	Tree	Fever Fever Malaria	Leaf Leaf Leaf	Decoction Decoction Decoction	Oral Oral Oral
	*Khaya senegalensis* A. Juss. (K008)	Mahogany (Akuapem/Krobo)	3.3	Tree	Infertility Male infertility	Bark Leaf	Decoction Decoction	Oral Oral

Menispermaceae	*Sphenocentrium jollyanum* Pierre (K026)	Kramaoti (Akuapem)	1.1	Herb	Diabetes	Whole plant	Decoction	Oral

Moringaceae	*Moringa oleifera* Lam. (A007)	Moringa	3.3	Tree	Blood tonic Pruritus Jaundice	Leaf Leaf Leaf	Decoction Decoction Decoction	Oral Oral Oral

Myrtaceae	*Psidium guajava* L. (K028)	Aguava (Akuapem/Krobo)	2.2	Shrub	Diarrhoea	Root	Decoction	Oral

Rutaceae	*Citrus sinensis* Pers. (K030)	Anka (Akuapem)/Kpeta (Krobo)	1.1	Tree	Constipation	Leaf and fruit	Infusion	Oral
	*Zanthoxylum leprieurii* Guill. & Perr. (K029)	Okanto (Akuapem)/Oyaa (Krobo)	2.2	Shrub	Sexual weakness Stroke	Leaf Root	Decoction Decoction	Oral Oral/Topical

Sapindaceae	*Lecaniodiscus cupanioides* Planch. (K031)	Unknown	1.1	Shrub	Stomach ulcer	Leaf	Decoction	Oral
	*Paullinia pinnata *L. (A002)	Tuatin (Twi) Detsemamu (Krobo)	6.5	Herb	Miscarriage Stomach ulcer Stroke HIV/AIDS Bone fracture	Leaf Leaf Leaf Leaf Leaf	Decoction Infusion Decoction Decoction Infusion	Oral Oral Oral Oral Oral/Rectal

Sapotaceae	*Aningeria altissima* (A. Chev.) Aubrév. (K033)	Asanfena (Twi)	2.2	Shrub	Stops bleeding	Leaf and bark	Decoction	Oral
	*Malacantha alnifolia* Pierre (K032)	Unknown	2.2	Shrub	Miscarriage	Leaf	Decoction	Oral

Solanaceae	*Physalis angulata* L. (K034)	Totoa (Krobo)	1.1	Herb	Cancer	Whole plant	Infusion	Oral/Topical
	*Solanum melongena* L. (A003)	Unknown	3.3	Shrub	Anaemia	Fruit	Infusion	Oral

**Table 3:** Information on considerations on factors of place and time during harvesting of medicinal plants by healers in some communities in southern Ghana.

Place/time	Factors/variables	Number of healers	Percentage of healers
Elevation	Lowland	44	97.8
	Highland	1	2.2
	Unimportant	0	0

Habitat	Wild	20	44.4
	Home garden	6	13.3
	Degraded area	16	35.6
	Unimportant	3	6.7

Seasonality	Wet season	9	20.0
	Dry season	3	6.7
	Both	30	66.7
	Unimportant	3	6.7

Soil type	Loam soil	34	75.6
	Sandy soil	8	17.7
	Clay soil	0	0
	Unimportant	3	6.7

Time of day	Morning	26	57.8
	Evening/night	0	0
	Afternoon	2	4.4
	Anytime	13	28.9
	Unimportant	4	8.9

Topography	Steep slope	0	0
	Gentle slope	4	8.8
	Flat land	41	91.1
	Unimportant	0	0

Vegetation type	Forest	17	37.8
	Savanna	2	4.4
	Forest-savanna mosaic	23	51.1
	Unimportant	3	6.6
